RETRACTED

# 17β-estradiol binding to ERα promotes the progression of prolactinoma through estrogen-response element-induced CaBP-9k up-regulation

**DOI:** 10.1042/BSR20191330

**Published:** 2020-01-14

**Authors:** Jun Liu, Hao Han, Wenpeng Lu, Gaoyang Fan

**Affiliations:** Department of Neuro Surgery, Jining No.1 People’s Hospital of Jining City Shandong Province, Jining City 272000, Shandong Province, China

**Keywords:** 17β-estradiol (E2), CaBP-9k, ERα, ERE, prolactinoma

## Abstract

17β-estradiol (E2) is considered to be an important instigator of prolactinoma, and can positively regulate the expression of calbindin-D9k (CaBP-9k) which contains an estrogen responsive element (ERE) via estrogen receptors (ERs). However, the detailed mechanism of E2 in promoting CaBP-9k expression and their roles in prolactinoma progression remain unclear. Here, we aimed to characterize it. The luciferase gene reporter assay with luc-ERE transfection showed that E2 treatment significantly enhanced the transcriptional level of CaBP-9k, whereas CaBP-9k activity was reduced when GH3 and MMQ cells were treated with AZD9496, an antagonist of ERα. E2 treatment increased the protein expressions of CaBP-9k and ERα but not ERβ, whereas this effect was also abolished when cells were treated with AZD9496. Besides, immunoprecipitation (IP) and immunofluorescence assays demonstrated that CaBP-9k could directly interact with ERα not ERβ, and Chromatin IP (ChIP) assay showed that ERα could bind to ERE of the CaBP-9k promoter. Moreover, cell counting kit-8 (CCK-8) and flow cytometry assays showed that E2 treatment significantly enhanced cell viability and inhibited cell apoptosis, but these effects were all abolished when ERα was down-regulated by short hairpin RNA (shRNA) or inhibited by AZD9496, as well as CaBP-9K suppression in both GH3 and MMQ cell lines. Taken together, these findings indicated that E2 stimulation promoted prolactin cell proliferation and inhibited cell apoptosis through ERα-induced CaBP-9k up-regulation, which then accelerated the advanced progression of prolactinoma.

## Introduction

The prolactin-secreting pituitary adenoma (prolactinoma) is the most common pituitary tumor, with an incidence of approximately 27 cases per million annually [1]. Although it has low incidence rate, prolactinoma is the most common pathologic reason for irregular menses, galactorrhea and infertility especially in young women [2]. Therefore, it is urgent to comprehensively inquire the mechanism underlying prolactinoma.

Estrogen receptors (ERs) are nuclear steroid hormone receptors and widely exist in normal pituitary tissues [3]. Although knowledge of the pathogenesis of prolactinoma is limited, estrogens are considered to be an important instigator in the progression of prolactinoma. In either male or female Fisher 344 rats, long-term administration of estrogens can lead to lactotroph hyperplasia or adenomas [4], which is now considered as a common method to build the *in vivo* prolactinoma model. Women accepting estrogens contraceptive have higher prolactinoma incidence with higher prolactin level [5]. In addition, it is well documented that binding to ERs, ERα and/or ERβ is the main mechanisms for estrogens activation [6,7]. However, the mechanisms underlying estrogens in accelerating the progression of prolactinoma still remain largely unknown.

RETRACTED

Calbindin-D9k (CaBP-9k) is encoded in humans by the S100G gene and is a vitamin D-dependent calcium binding protein. It is reported that CaBP-9k expression can be increased following 17β-estradiol (E2) or E-BSA (membrane impermeable E2-conjugated with BSA) administration in GH3 cells [8,9], a mouse pituitary gland tumor cell line [10]. Consistently, in our previous study [11], we showed that E2 treatment increased the expression of CaBP-9k at both mRNA and protein levels, together with enhanced interaction between CaBP-9k and ERα proteins. However, the increased expression of CaBP-9k caused by E-BSA was neutralized when ER was blocked by ICI182780 [8], a selective estrogen antagonist on both ERs, suggesting that E2 positively regulates CaBP-9k expression in an ER-dependent manner in GH3 cells. However, the molecular mechanism underlying E2 to up-regulate CaBP-9k is still not completely clear. It is reported that CaBP-9k promoter contains an estrogen responsive element (ERE) and a progesterone responsive element (PRE), which are known to regulate CaBP-9k transcription in rat uterus [12,13]. We speculated that ERE might be a possible mechanism underlying estrogens to regulate CaBP-9k expression.

As a result, the present study was performed with two main purposes, one was to explore whether estrogens positively regulate CaBP-9k expression through ERE, and the other was to elucidate the effects of E2/ERα/CaBP-9k axis in the progression of prolactinoma.

## Materials and methods

### Cell culture and treatment

Rat pituitary adenoma cell lines MMQ and GH3 were obtained from BeNa Culture Collection (Beijing, China) and were cultured in F-12K Medium (Gibco, Thermo Fisher Scientific, MA, U.S.A.), supplemented with 2.5% fetal bovine serum (FBS) (Gibco) and 15% horse serum (HyClone, UT, U.S.A.) in a humidified atmosphere at 37°C with 5% CO_2_.

Cells were incubated with 0.1, 1 or 10 nM of E2 (Sigma–Aldrich Corp, MO, U.S.A.) dissolved in 0.1% (vol/vol) DMSO for 24 h. To block ERs, MMQ or GH3 cells were treated with 1 μM of ICI182780 (Tocris, MO, U.S.A.), an ER antagonist, for 30 min prior to E2 administration. To specially block ERα, MMQ or GH3 cells were treated with 300 nM of AZD9496 (No. HY-12870, MedChemExpress, Shanghai, China), an ERα antagonist, for 1 h prior to E2 administration.

RETRACTED

### RNA interference

Short hairpin RNAs (shRNAs) used to silence ERα (sh-ERα; No. TL510613) or (sh-CaBP-9k, No. TL709169), and the negative control vectors (sh-NC) were purchased from OriGene (Beijing, China).

### Western blotting analysis

Total protein was obtained from cells using RIPA buffer containing phosphatase and protease inhibitors (Beyotime Biotechnology, Shanghai, China). After quantification, 30 μg proteins from each sample were loaded into and separated by 10% SDS/PAGE, and subsequently transferred on to the polyvinylidene difluoride membranes (PVDF, Thermo Fisher Scientific). Next, the membrane was blocked with 5% non–fat milk for 1 h at room temperature, and incubated with the primary antibodies CaBP-9k (No. sc-74462, Santa Cruz, CA, U.S.A.), ERα (No. ab32063, Abcam, MA, U.S.A.), ERβ (No. sc-53494, Santa Cruz) or GAPDH (Proteintech, Hubei, China) overnight at 4°C. Subsequently, the membranes were incubated with the corresponding secondary antibodies (AmyJet Scientific Inc., Hubei, China) at room temperature for 1 h. Bound antibodies were detected by gel document system using enhanced chemiluminescence (ECL) reagent (Millipore, MA, U.S.A.). ImageJ software (National Institutes of Health, Bethesda, MD, U.S.A.) was used to quantify protein expression levels. GAPDH was served as an internal reference to normalize protein expression.

### Immunoprecipitation

The immunoprecipitation (IP) of CaBP-9k was performed using Dynabeads Protein A (Invitrogen, CA, U.S.A.) in accordance with the manufacturer’s protocol. Briefly, cells were lysed in 5 ml lysis buffer (50 mM Tris/HCl, pH 7.5, 200 mM NaCl, 0.5% Nonidet P40, protease inhibitor cocktail) for 30 min at 4°C. After 1 h of incubation with 50 μl protein A, the supernatants were incubated with anti-CaBP-9k antibody (No. sc-74462, Santa Cruz) at 4°C overnight. Next, the beads were washed with Western/IP lysis buffer for five times, followed by being resuspended in SDS/PAGE loading buffer (Beyotime, Jiangsu, China). The immune complex was then submitted to Western blotting analysis with antibodies against ERα (No. ab32063, Abcam) or ERβ (No. sc-53494, Santa Cruz).

### Chromatin IP assay

Chromatin IP (ChIP) assay used to evaluate the interaction between ERα and ERE located in CaBP-9k promoter was performed as previously described [14]. The cross-linked chromatins were immunopreciptated with anti-ERα antibody (No. ab32063, Abcam). The enrichment of the specific amplified region was analyzed by real-time quantitative PCR (RT-PCR). The primers for amplifying the fragments of the ERE in CaBP-9k promoter are as follows: forward-5′-CTCTTCTTCGACCCAGCCTTGC-3′ and reverse-5′-GGAGGCAGCGAGAAAGCG-3′.

RETRACTED

### Immunofluorescence

GH3 cells grown on coverslips were washed three times with PBS, followed by fixation in 4% paraformaldehyde for 10 min, permeation with 0.1% Triton X-100, and blockage with 5% goat serum diluted in PBS for 1 h. Next, the cells were co-incubated with anti-CaBP-9k (No. sc-74462, Santa Cruz) and anti-ERα (No. ab32063, Abcam) antibodies overnight at 4°C and then incubated with the Alexa Fluor® 488 Conjugate and Alexa Fluor® 568 Conjugate fluorescent second antibodies (Cell Signaling Technology, MA, U.S.A.) at room temperature for 1 h in the dark. Finally, the cells were stained with DAPI solution (Solarbio, Beijing, China) for 5 min and covered with antifade mounting medium. The expressions of CaBP-9k and ERα were analyzed by using a fluorescence microscope (Olympus Confocal FV100 Microscope).

### Luciferase gene reporter assay

To analyze the effect of E2/ERα axis on the transcriptional regulation of CaBP-9k, luciferase report vector coding ERE which is located in CaBP-9k promoter was constructed by GenePharm (Shanghai, China) and named as ERE-Luc. After being treated with E2 (1 nM) together with 1 μM of ICI182780, MMQ and GH3 cells were transfected with ERE-Luc using the Lipofectamine 2000 reagent (Invitrogen). The luciferase activity was measured by using the luciferase assay system (Promega, Madison, WI, U.S.A.) according to the manufacturer’s instructions.

### Cell counting kit-8 assay

MMQ or GH3 cells (2000 cells for each well) were seeded in 96-well plates and incubated at 37°C overnight, then cells were subjected to different treatments including shRNAs, E2 or AZD9496. After 48 h of the treatment, 10 μl of cell counting kit-8 (CCK-8) reagent (Dojindo, Japan) was added into each well and incubated for another 4 h at 37°C. The optical density (OD) levels at 450 nm were measured using a microplate reader.

### Flow cytometry

After 48 h of treatments with shRNAs, E2 or AZD9496, MMQ and GH3 cells were collected and washed with PBS once. Then, cells were dyed with the Annexin V-FITC/PI kit (BD Bioscience, San Diego, CA, U.S.A.) referring to the manufacturer’s descriptions. The fluorescent signal was measured by flow cytometry within 1 h of staining. Cells in FITC^−^/PI^−^ quadrant were living cells, FITC^+^/PI^−^ were early apoptotic cells and FITC^+^/PI^+^ were late apoptotic cells.

### Statistical analysis

Data were recorded from as least three independent experiments and were expressed as mean ± standard deviation (SD). SPSS 22.0 software (Chicago, IL, U.S.A.) was used to performed data analysis with *t* test or one-way analysis of variance (ANOVA) for comparisons between two groups or multiple groups. A *P-*value less than 0.05 was considered to be statistically significant.

RETRACTED

## Results

### E2 positively regulates the transcriptional level of CaBP-9k through ER-mediated ERE activation in CaBP-9k promoter

To explore the mechanism of E2 to increase CaBP-9k expression, we first carried out the luciferase gene reporter assay using ERE-Luc vector. The results showed that E2 treatment significantly increased the transcriptional level of CaBP-9k, whereas this effect was abolished when ERs were blocked by ICI182780 in both MMQ and GH3 cells (Figure 1A,B). This result indicated that E2 up-regulated CaBP-9k expression in an ER-induced ERE activation manner.

**Figure 1:** E2 promoted the transcription of CaBP-9k through ERs-induced ERE activation MMQ and GH3 cells were treated with E2 (1 nM) or E2 + ICI182780 (1 μM) and transfected with luc-ERE, then (**A,B**) the luciferase reporter gene assay was carried out to evaluate the effects of E2 and ERs on CaBP-9k transcription (*P<0.05, compared with NC group, ^#^*P*<0.05, compared with E2 group).

### E2 increases CaBP-9k expression through ERα

Next, we further explored which one of the two ERs was involved in the mechanism of E2 in increasing CaBP-9k expression. Compared with the control group, E2 treatment significantly increased the protein expression levels of ERα and CaBP-9k in GH3 and MMQ cells in a dose-dependent manner, whereas showed no obvious influence in ERβ expression (Figure 2A,B). As 1 nM E2 significantly increased CaBP-9k and ERα expression in both cell lines, we chose 1 nM E2 for further study. To further reveal the effects of ERα on E2-induced CaBP-9k up-regulation, we used AZD9496 to suppress ERα, and the results showed that the increased expressions of ERα and CaBP-9k induced by E2 treatment were neutralized after GH3 and MMQ cells were treated with AZD9496 (Figure 2C,D). These results demonstrated that E2 up-regulated CaBP-9k expression through ERα but not ERβ.

**Figure 2:** E2 increased CaBP-1 expression through ERα (**A,B**) MMQ and GH3 cells were treated with 0, 0.1, 1 and 10 nmol/l E2 for 24 h, then the cells were collected and submitted to (A,B) Western blotting assay to test the protein expression levels of CaBP-9k, ERα and ERβ (*P<0.05). (**C,D**) GH3 and MMQ cells were treated with 300 nM AZD9496 for 1 h prior to 1 nM E2 treatment, then the cells were harvested and subjected to Western blotting to test the protein expressions of CaBP-9k, ERα and ERβ (*^,+^*P*<0.05, compared with NC group; ^#^P<0.05, compared with E2 group).

RETRACTED

### ERα directly binds to the ERE in CaBP-9k promoter

To further study the mechanism of E2/ERα in promoting CaBP-9k expression, we carried out IP and immunofluorescence assays to evaluate the interaction between ERs and CaBP-9k proteins. IP assay demonstrated that CaBP-9k could directly binding to ERα but not ERβ, and E2 treatment significantly enhanced their interaction (Figure 3A). Immunofluorescence results showed that there was co-location of ERα and CaBP-9k proteins in nucleus (Figure 3B). In addition, the results from ChIP assay also demonstrated that ERα not ERβ could directly combine with the ERE in CaBP-9k promoter (Figure 4). Overall, these discoveries demonstrated that ERα could directly interact with CaBP-9k through binding to ERE.

**Figure 3:** ERα could bind to CaBP-9k protein (**A**) IP assay was carried out to analyze the interaction between CaBP-9k protein and ERα/ERβ protein in GH3 cells. (**B**) The subcellular location of CaBP-9k and ERα proteins in GH3 cells were determined by immunofluorescence.

**Figure 4:** ERα could bind to the ERE of CaBP-9k promoter ChIP assay was performed to analyze the interaction between ERE and ERα or ERβ.

### E2 treatment facilitates the proliferation and inhibits the apoptosis of GH3 and MMQ cells in an ERα-dependent manner

Next, we investigated the effects of E2/ERα/CaBP-9k axis in the progression of prolactinoma. Infection with sh-ERα2 and sh-ERα3 significantly decreased ERα expression and sh-ERα2 showed the highest knockdown efficiency (Figure 5A) and was chosen for the following experiments. E2 treatment obviously enhanced cell viability of GH3 and MMQ cells, whereas this effect was impaired when ERα was silenced by sh-ERα or inhibited by AZD9496 (Figure 5B,C). In addition, the effect of E2 treatment on cell apoptosis repression was also weakened by sh-ERα or AZD9496 treatment (Figure 5D,E), as well as the increased expression of CaBP-9k induced by E2 treatment (Figure 5F–H). The above results demonstrated that E2 treatment promoted prolactinoma progression in an ERα-dependent manner.

**Figure 5:** E2 facilitated the proliferation and inhibited the apoptosis of GH3 and MMQ cells through ERα (**A**) The knockdown efficiency of sh-ERα in GH3 and MMQ cells was determined by Western blotting assay. MMQ and GH3 cells were treated with E2, E2+AZD9496, or E2+sh-ERα, then cells were collected for the following assays. (**B,C**) CCK-8 assay used for cell viability detection. (**D,E**) Flow cytometry used for cell apoptosis detection. (**F,H**) Western blotting analysis used for detection of the protein expression of CaBP-9k (*P<0.05, compared with NC group; ^#^*P*<0.05, compared with E2 group).

RETRACTED

### E2 treatment promotes the proliferation and inhibits the apoptosis of GH3 and MMQ cells through increasing CaBP-9k expression

We then applied the shRNAs to down-regulate CaBP-9k expression to elucidate CaBP-9k roles in E2-mediated prolactinoma progression. The shRNA-1 targeting CaBP-9k gene presented with the highest knockdown efficiency among the three shRNAs (Figure 6A) and was chosen for the following assays. Down-regulation of CaBP-9k obviously rescued the effects of E2 treatments on cell viability promotion (Figure 6B,C) and apoptosis inhibition (Figure 6D,E) in both MMQ and GH3 cell lines. These results demonstrated that E2 treatment accelerated the progression of prolactinoma via increasing CaBP-9k expression.

**Figure 6:** E2 treatment facilitated the proliferation and inhibited the apoptosis of GH3 and MMQ cells through increasing CaBP-9k expression (**A**) The knockdown efficiency of sh-CaBP-9k was determined by Western blotting assay in both MMQ and GH3 cell lines. Then, MMQ and GH3 cells were treated with E2, sh-CaBP-9k or E2+sh-CaBP-9k and then were submitted to the following assays. (**B,C**) CCK-8 assay was used to detect cell viability. (**D,E**) Flow cytometry was performed to detect cell apoptosis (*P<0.05, compared with NC group, ^#^*P*<0.05, compared with E2 group).

## Discussion

E2 is identified to be an important instigator of prolactinoma [15], suggesting that E2 might be a potent therapeutic target for prolactinoma. Evidence has indicated that E2 increases CaBP-9k expression through ERs [11,16]. However, it is not entirely clear that the detailed mechanism underlying E2 in promoting CaBP-9k expression and their role in the development of prolactinoma. The present study demonstrated that E2 positively regulated CaBP-9k expression through activation of ERE region in CaBP-9k promoter in an ERα-dependent manner, which then accelerated the proliferation and inhibited the apoptosis of pituitary cells.

Estrogens are strongly implicated in regulating secondary sexual characteristics, inflammatory responses and the development of prolactinoma and breast cancer via binding to ERs, ERα and/or ERβ [17,18]. ERs is mainly expressed in nucleus [19], with a small amount of it expressed in plasma membrane [20]. Estrogens can directly enter the nucleus and bind to the nuclear ERs, regulating gene transcription through the specific binding sites of ERE in their target genes, which is considered as the genomic pathway. Once combined with the membrane ERs, estrogens activate the G proteins and induce or modulate downstream pathways activation, such as extracellular regulated kinase (ERK) and protein kinase B (Akt) signalings [11,21], which is considered as the non-genomic pathway. Interestingly, ERα differs from ERβ in certain aspects. For example, in the uterus, ERα is expressed in the epithelial cells, glandular epithelial cells, and stromal cells while ERβ is expressed in glandular epithelial cells [22]. Notably, uterine CaBP-9k was up-regulated when the immature female Sprague–Dawley rats were given propyl pyrazole triol (PPT, an ERα-selective ligand) in a dose- and time-dependent manner, whereas CaBP-9k expression showed no significant alteration after diarylpropionitrile (DPN, an ERβ-selective ligand) treatment; in addition, the increased expression of CaBP-9k was completely abolished by ICI182780, an antagonist of ERs, indicating that CaBP-9k expression is under the regulation of ERs [16]. In the present study, we observed that ERα down-regulation with shRNA infection or inhibition with AZD9496 abrogated the role of E2 in CaBP-9k expression promotion. Furthermore, the present study also demonstrated that E2 treatment increased ERα expression, whereas showed no obvious influence in ERβ expression, and CaBP-9k protein interacted directly with ERα but not ERβ. All suggesting that E2 increased CaBP-9 expression in an ERα-dependent manner.

RETRACTED

Evidences have shown that ligand-activated ERs positively or negatively modulate gene transcription via binding to the specific ERE within their target genes [23]. For example, E2 was shown to increase prolactin transcription through ERE which is located upstream of the 5′-regulatory region of prolactin [24,25]. Coincidentally, CaBP-9k promoter also contains the minimal ERE at nucleotides +51 to +61, which was able to bind to ERα [26]. In this view, we performed luciferase gene reporter assay to clarify the molecular mechanism underlying E2-induced CaBP-9k up-regulation. The results showed that E2 increased CaBP-9k transcriptional activity through ERE, whereas this effect was abolished when ERs were inhibited; besides, ChIP assay showed that ERα not ERβ could bind to the ERE region of CaBP-9k gene, implying that E2 activated CaBP-9k transcription through a binding between ERα and ERE.

After clarification of the mechanism of E2 in CaBP-9k expression, we also explored the function of E2/ERα/CaBP-9k axis in the progression of prolactinoma. The results showed that repression of ERα or CaBP-9k significantly impaired the effects of E2 on cell viability enhancement and cell apoptosis reduction. These results indicated that ERα and CaBP-9k exerted an important role in E2-mediated prolactinoma progression, which was consistent with a previous study [27]. Moreover, Cenni and Picard [28] and El-Tanani and Green [29] also revealed that ERα promoted the production of growth factors or cytokines to facilitate MMQ cell proliferation and prolactin secretion without exogenous E2 stimulation.

RETRACTED

In conclusion, the current study reveals that E2 treatment promotes prolactin cell proliferation and inhibits cell apoptosis through ERα-induced CaBP-9k up-regulation, resulting in the advanced progression of prolactinoma. The present study may provide a potent target of ERα/CaBP-9k for prolactinoma treatment.

## Abbreviations

CaBP-9k: calbindin-D9k
ChIP: chromatin immunoprecipitation
ERE: estrogen responsive element
ER: estrogen receptor
E2: 17β-estradiol
GAPDH: glyceraldehyde-3-phosphate dehydrogenase
IP: immunoprecipitation
PI: propidium iodide
PIPA: radio-immunoprecipitation assay
shRNA: short hairpin RNA
